The article "Acute and sub-acute oral toxicity of Dracaena cinnabari resin methanol extract in rats" was published in 2018. Journal: BMC Complement Altern Med.

# Acute and sub-acute oral toxicity of *Dracaena cinnabari* resin methanol extract in rats

**DOI:** 10.1186/s12906-018-2110-3

**Published:** 2018-02-05

**Authors:** Nashwan Abdullah Al-Afifi, Aied Mohammed Alabsi, Marina Mohd Bakri, Anand Ramanathan

**Affiliations:** 1 Department of Oral and Craniofacial Sciences, Faculty of Dentistry, University of Malaya, 50603 Kuala Lumpur, Malaysia; 2 Department of Oral Biology and Biomedical Sciences, Faculty of Dentistry, MAHSA University, 42610 Jenjarom, Selangor Malaysia; 3 Department of Oral & Maxillofacial Clinical Sciences, Faculty of Dentistry, University of Malaya, Kuala Lumpur, 50603 Malaysia; 4 Oral Cancer Research and Coordinating Centre, Faculty of Dentistry, University of Malaya, Kuala Lumpur, 50603 Malaysia

**Keywords:** DC resin methanol extract, Acute oral toxicity, Sub-acute oral toxicity, Histopathology, Hematological parameters, Biochemical parameters

## Abstract

**Background:**

*Dracaena cinnabari* (DC) is a perennial tree that located on the Southern coast of Yemen native to the Socotra Island. This tree produces a deep red resin known as the Dragon’s blood, the Twobrother’s Blood or Damm Alakhwain. The current study performed to evaluate the safety of the DC resin methanol extract after a single or 28 consecutive daily oral administrations.

**Methods:**

In assessing the safety of DC resin methanol extract, acute and sub-acute oral toxicity tests performed following OECD guidelines 423 and 407, respectively, with slight modifications. In acute oral toxicity test, DC resin methanol extract administered to female Sprague Dawley rats by oral gavage at a single dose of 300 and 2000 mg/kg body weight. Rats observed for toxic signs for 14 days. In sub-acute oral toxicity test, DC resin methanol extract administered to the rats by oral gavage at 500, 1000, and 1500 mg/kg body weight daily up to 28 days to male and female Spradgue Dawley rats. The control and high dose in satellite groups were also maintained and handled as the previous groups to determine the late onset toxicity of DC resin methanol extract. At the end of each test, hematological and biochemical analysis of the collected blood were performed as well as gross and microscopic pathology.

**Results:**

In acute oral toxicity, no treatment-related death or toxic signs were observed. It revealed that the DC resin methanol extract could be well tolerated up to the dose 2000 mg/kg body weight and could be classified as Category 5. The sub-acute test observations indicated that there are no treatment-related changes up to the high dose level compared to the control. Food consumption, body weight, organ weight, hematological parameters, biochemical parameters and histopathological examination (liver, kidney, heart, spleen and lung) revealed no abnormalities. Water intake was significantly higher in the DC resin methanol extract treated groups compared to the control.

**Conclusion:**

This study demonstrates tolerability of DC resin methanol extract administered daily for 28 days up to 1500 mg/kg dose.

**Electronic supplementary material:**

The online version of this article (10.1186/s12906-018-2110-3) contains supplementary material, which is available to authorized users.

## Background

Medicinal plants are used worldwide to treat many diseases, and new drugs continue to be developed through research from these plants [1]. Medicinal plant preparations can be formulated into many forms including liquids, and they have been used worldwide for many years [2]. The use of a medicinal plant for the treatment of disease without the scientific foundation to adequately support conclusions of safety and efficacy can be potentially dangerous as well as useless. In addition, misuse of these medicinal plants may cause serious toxicity for humans [3]. As chemical compositions of the medicinal plant are complex, some moderate to severe side effects may arise from the use of herbal medicines. Therefore, it is important to establish medicinal plant safety through the use of well-controlled and validated scientific toxicity studies or protocols [4].

Toxicological studies subjected to make a decision about whether a new drug should be accepted for clinical use or not [5]. Toxicity study gives information on toxic doses and therapeutic indices of drugs and xenobiotic [6]. The outcome of the toxicity study in animals is vitally needed to determine the safety of medicinal plants if they are found to be suitable for development into pharmacological products. In addition, to determine the appropriate dose for long-term toxicity tests and to determine the affected organs at the end of the treatment, the toxicity test is achieved [7]. It is a scientific, ethical and regulatory requirement that before any potential new medicine administered to humans, its safety must be investigated in animals to define safe human doses [8].

*Dracaena cinnabari* (DC) is a perennial tree located on the Southern coast of Yemen native to the Socotra Island. This tree produces a deep red resin which called the Dragon’s blood or the Twobrother’s Blood [9]. DC belongs to Agavaceae family, which is commonly known as Damm Alakhwain in Yemen [10]. It is a large, single-trunked tree with height up to 10 m and smooth grey bark. Branches with sausage-shaped sections form an umbrella-shaped crown [11]. DC tree populations on Socotra do not regenerate to a significant extent, and their age structure indicates overmaturity [12]. The red “dragon’s blood” resin of the DC tree exudes from fissures and wounds in the bark or branches [1]. People in Socotra used the resin from DC for dying wool, glue pottery, breath freshener, to decorate a pottery and houses and even as lipstick [13]. In addition, DC resin has been a famous traditional medicine since ancient times in many cultures. It is used as an astringent for treating diarrhea and dysentery as well as an antiseptic, haemostatic and as an antiulcer remedy [1, 10, 14, 15]. Phytochemical studies of DC resin have led to the isolation of several active compounds belonging to the flavanoids, homoisoflavonoids, chalcones, sterols and terpenoids. Some homoisoflavonoids and chalcones isolated from the DC resin exhibited a strong antioxidant activity [16]. The presence of flavonoids reported contributing in anti-inflammatory activities of methanol extract of DC resin [17]. The chemical constituents of DC resin have been reviewed by D Gupta, B Bleakley and RK Gupta [1]. The methanolic extract of DC resin has been reported to exert an antiviral activity against Herpes simplex and Human influenza viruses [18]. DC resin is showing enormous potential interaction with antimicrobial [19] and antioxidants activities [10, 20] and considered as good source of food preservative due to its inhibitory effect on various foodborne pathogens [20]. A methanol extract of DC resin exhibited a non-specific inhibition of the parasites related to high cytotoxicity [21].

Despite its wide uses, no study has been done to know about its oral toxicity which in turn will provide proper safety information regarding DC resin and to define safe human doses. Thus, the aim of the current study is to evaluate the safety of the DC resin methanol extract after a single or 28 consecutive daily oral administrations.

## Methods

### Preparation of *Dracaena cinnabari* (DC) resin extract

The resin of DC collected from Socotra Island (Yemen) in May 2013. The plant samples were identified and authenticated by Environmental Protection Authority of Yemen. A voucher specimen of the resin (DC/2013-8/122) has been deposited at the herbarium of department of Pharmacognosy, Faculty of Pharmacy, University of Sana’a, Yemen.

DC resin was ground into powder form using an electrical blender to ease the extraction process. 50 g of the powdered resin of DC placed into a 1 L conical flask then macerated with methanol (500 ml methanol was added in, where 1 g of dried and ground DC is to 10 ml methanol) in the ratio of (1:10). Methanol has high polarity and thus greater efficacy towards the extraction of polar phytochemicals such as phenolics and flavonoids [22]. The conical flask was left at room temperature for approximately 3 days on a shaker at 100 rpm. The resultant extract filtered through a fine muslin cloth, and then a filter paper Whatman (Grade 1-Circles, 150 mm) was used to remove the crude part. For separating the methanol from the extract, Eyela rotary evaporator used under reduced pressure at 40 °C which produced a gummy red resin extract. After that, a freeze dryer was used to provide 28.0 g of a dry powder extract. The extract was then wrapped with aluminum foil to prevent a photo-oxidation that might be occurred and was stored at 4 °C until used. This methanol extract dissolved in (10% DMSO) before use.

### Experimental animals

Female and male Sprague Dawley (SD) rats were used for the acute and sub-acute oral toxicology tests. Nine rats (females) were used in an acute oral toxicity test, whereas 60 rats (30 males and 30 females) used in sub-acute oral toxicity test (the repeated dose 28 day). The toxicity tests were carried out according to Organization for Economic Cooperation and Development (OECD) test guideline, i.e., OECD Guideline 423 for the acute oral toxicity test [23] and OECD Guideline 407 for the sub-acute oral toxicity test [24] with slight modifications. The rats were obtained from the Animal Experimental Unit, Faculty of Medicine, University of Malaya, Kuala Lumpur. SD rats (8-10 weeks) weigh between 235 ± 15 g were used. Prior to the start of the experiment, body weight of animals was recorded individually for calculating proper treatment dosage. The volume was adjusted depending on the body weight of the rat using 10 ml/kg as this is the normal volume to be used in the rat as mentioned elsewhere [25, 26]. The female SD rats were nulliparous and non-pregnant. The SD rats were given standard rat pellets and reverse osmosis (RO) water ad libitum. They were acclimatised to laboratory conditions for 7 days before the experiments and housed in groups of three for acute oral toxicity and in groups of five for sub-acute oral toxicity. The rats were maintained at a room temperature of 24 °C, with a 12 h light/dark cycle. Protocols approved by the Institutional Animal Care and Use Committee (IACUC), Faculty of Medicine, University of Malaya, Malaysia (Ethics No. 2014-02-14/OBBS/R/NAA). The endpoint of all rats considered when around 20% of body weight loss has been shown.

### Acute oral toxicity

The DC resin methanol extract was administered to the female rats under overnight fasting by using oral gavage in a volume of 10 ml/kg body weight.

Nine female SD rats were randomly divided into 3 groups of 3 rats each as mentioned previously [27]. The started dose at 300 mg/kg body weight of DC resin methanol extract that dissolved in 10% DMSO administered to the group 1. The rats were observed for general behavioural changes; symptoms of toxicity and mortality after treatment for the first 4 h, then over a period of 48 h. Group 2 was administrated sequentially at 48-h intervals with the next higher dose 2000 mg/kg body weight of DC resin methanol extract that dissolved in 10% DMSO when there were no signs of toxicity or mortality showed in group 1 after 48 h of treatment. In parallel, group 3 added and treated with vehicle (10% DMSO) to establish a comparative negative control group according to the OECD guideline [23]. All animals observed at least once during the first 30 min in the first 24 h with great consideration given for the first 4 h following vehicle or DC resin methanol extract administration and then once a day for 14 days. This observation was done to check the onset of clinical or toxicological symptoms according to the OECD guideline [23]. All observations included changes in skin and fur, eyes and mucous membranes and behavioral pattern were systematically recorded and maintained with an individual record. In addition, consideration was given for observations of convulsions, tremors, diarrhea, salivation, lethargy, sleep, coma and mortality. The food consumption and water intake recorded daily. The body weights of animals recorded shortly before the administration of the tested substance and at the end of each week. The percentage of body weight change calculated according to the following equation:

$$ \frac{\mathrm{Body}\kern0.5em \mathrm{weight}\kern0.5em \mathrm{at}\kern0.5em \mathrm{the}\kern0.5em \mathrm{end}\kern0.5em \mathrm{of}\kern0.5em \mathrm{each}\kern0.5em \mathrm{week}\hbox{-} \mathrm{initial}\kern0.5em \mathrm{body}\kern0.5em \mathrm{weight}}{\mathrm{Initial}\kern0.5em \mathrm{body}\kern0.5em \mathrm{weight}}\times 100 $$

### Sub-acute oral toxicity (repeated dose 28-day oral toxicity)

The SD rats were randomly divided into six groups of 10 rats each (*n* = 10/group, 5 males and 5 females) as mentioned elsewhere [28]. Four groups were administered daily with DC resin methanol extract at different concentration dissolved in 10% DMSO and two groups administered with the vehicle by using oral gavage. Group 1 received vehicle (10% DMSO) and served as control. Groups 2, 3 and 4 received doses of DC resin methanol extract at 500, 1000 and 1500 mg/kg body weight, respectively. The 5th and 6th groups namely satellite groups added to determine the reversibility or recovery from toxic effects of the test material and given the vehicle (10% DMSO) and the top dose of DC resin methanol extract 1500 mg/kg body weight, respectively. They were handled as the previous groups. The test material was administered orally (gavage) once daily for 28 consecutive days. The satellite groups were scheduled for follow-up observations for the next 14 days without a vehicle or DC resin methanol extract administration.

Mortality, food consumption and water intake, as well as observation for general toxicity signs of the animals, were monitored and recorded daily throughout the study. The initial body weight of all the groups has been recorded before the tested material is administered and at the end of each week.

### Hematology and serum biochemistry

At the end of each experiment (at 15^th^ day for acute oral toxicity and at 29^th^ day for sub-acute oral toxicity tests except the satellite groups which were at 43^rd^ day), the rats generally anesthetized by intraperitoneal injection of 80 mg/kg of ketamine 100 mg/ml + 7 mg/kg of xylazine 100 mg/ml (Troy Laboratories PTY. Limited, Smithfield, Australia). Blood sample (5 ml) by cardiac puncture was collected using a disposable syringe. The blood kept in K2EDTA tube for analysing hematological parameters [haemoglobin (HGB), white blood cell (WBC), Neutrophil, Lymphocyte, Monocyte, Eosinophil and Basophil] and in Plain tubes for biochemical parameters [Urea, Creatinine, Albumin, Globulin, Total bilirubin, Conjugate Bilirubin, Alkaline phosphatase (ALP), Alanine transaminase (ALT) and Aspartate aminotransferase (AST)]. The blood sample that placed in a plain tube left for 15 - 20 min at room temperature to promote blood coagulation. The blood sample was centrifuged at 5000 rpm for 20 min at 4 °C; the serum obtained then analysed. Immediately, after blood collection, rats were sacrificed by cervical dislocation.

### Histopathological observation

Necropsy was done in acute and sub-acute oral toxicity tests groups of animals on day 15 and 29 respectively, and for the satellite groups, on day 43. After the blood collection, rats were sacrificed by cervical dislocation, and the vital organs (liver, kidney, heart, spleen and lung) removed through a midline incision in the Rat’s abdomen. The organs were cleaned of fat and blotted with clean tissue paper, and then weighed on balance. The relative organ’s weight (ROW) were calculated and recorded in proportion to the body weight according to the following equation:

$$ \mathrm{RWO}=\frac{\mathrm{Absolute}\kern0.5em \mathrm{organ}\kern0.5em \mathrm{weight}}{\mathrm{Body}\kern0.5em \mathrm{weight}\kern0.5em \mathrm{at}\kern0.5em \mathrm{sacrifice}}\times 100 $$

Samples from the vital organs (liver, kidney, heart, lung and spleen) of both acute and sub-acute oral toxicity tests were subjected to histopathological evaluation. They fixed in 10% buffered formalin, routinely processed and embedded in paraffin wax. Paraffin sections (5 μm) was cut on glass slides and stained with hematoxylin and eosin. An experienced pathologist who was unaware of the experimental groups to which each section belonged conducted the analysis. The slides were examined under a light microscope (Nikon E50i, Nikon Corporation, Japan) as mentioned elsewhere [29].

### Statistical analysis

Results expressed as a mean ± standard deviation. The differences between groups of acute and sub-acute toxicity tests determined by one-way analysis of variance (ANOVA) followed by Tukey multiple comparison test, and Student *t* test for satellite groups comparisons. Differences were considered significant at *p* < 0.05.

## Results

### General sign and behavioral analysis

Oral administration of DC resin methanol extract showed no treatment-related mortality in both sexes of rats for both acute and sub-acute oral toxicity tests throughout the study. Physical observation of the DC treated rats for both acute and sub-acute oral toxicity tests throughout this study indicated that none of them showed signs of toxic effects such as changes in skin and fur, eyes and mucous membrane, behavior pattern, tremors, salivation, diarrhea and coma. No gross or microscopic pathological abnormalities in all groups (acute and sub-acute oral toxicity tests) observed in any animals. Concerning the Globally Harmonized Classification System, DC resin methanol extract can be classified as Category 5 and this provides direct relevance for protecting animal and human health up to the high dose level that used in this study.

### Effect of DC extract on body weight, organ’s weight, food consumption and water intake in acute and sub-acute oral toxicity tests

A raw data of body weight, organ’s weight, food consumption and water intake, is available in the Additional file 1.

The body weight of the control and DC treated rats were as shown in Table 1 (A and B). There was a gradual increase in body weight of the control and DC treated groups in both acute and sub-acute oral toxicity tests. The percentage changes in body weight of the DC treated groups were not significantly different compared to the control rats as *p* > 0.05 (Table 1 A and B). In addition, there is no significant different has been shown in Satellite groups in both sexes with *p* > 0.05 (Table 2).

**Table 1:** (A and B) Percentage of body weight gain of rats in acute and sub-acute oral toxicity tests at each week

A	Acute oral toxicity					
	Sex	Control	DC 300 mg/kg	DC 2000 mg/kg		*P* value
0 day (g)	F (*n* = 3)	235.33 ± 5.03	250.00 ± 8.54	249.67 ± 9.61		
Week 1 (%)	F (*n* = 3)	5.82 ± 1.44	4.92 ± 1.62	4.15 ± 0.37		0.340
Week 2 (%)	F (*n* = 3)	8.65 ± 1.96	8.53 ± 1.59	7.37 ± 1.17		0.586
B	Sub-acute oral toxicity					
	Sex	Control	DC 500 mg/kg	DC 1000 mg/kg	DC 1500 mg	*P* value
0 day (g)	M (*n* = 5)	232.00 ± 4.70	223.40 ± 5.22	226.40 ± 5.13	229.80 ± 3.96	
	F (n = 5)	247.20 ± 6.14	233.40 ± 2.70	228.60 ± 8.02	232.20 ± 2.56	
Week 1 (%)	M (n = 5)	8.28 ± 0.91	8.56 ± 0.79	8.11 ± 1.15	8.61 ± 1.28	0.853
	F (n = 5)	5.03 ± 2.44	4.71 ± 1.09	5.44 ± 1.71	5.50 ± 2.21	0.907
Week 2 (%)	M (*n* = 5)	16.73 ± 1.03	16.37 ± 1.19	16.78 ± 0.83	16.09 ± 1.87	0.811
	F (*n* = 5)	7.53 ± 3.21	7.62 ± 2.09	7.27 ± 2.59	8.49 ± 2.30	0.889
Week 3 (%)	M (*n* = 5)	24.25 ± 2.13	24.17 ± 1.09	23.69 ± 1.64	23.48 ± 2.00	0.881
	F (*n* = 5)	11.42 ± 2.77	10.44 ± 2.82	10.55 ± 2.64	12.30 ± 3.20	.0715
Week 4 (%)	M (*n* = 5)	29.34 ± 2.70	28.55 ± 1.60	29.71 ± 2.08	29.75 ± 4.94	0.920
	F (*n* = 5)	13.83 ± 2.76	13.18 ± 2.24	13.36 ± 3.05	15.23 ± 2.94	0.649

Values expressed as a mean ± standard deviation. Sex (male, M and female, F)

*p-value less than 0.05, (*p* < 0.05) significant value

**Table 2:** Satellite group/ Percentage of body weight change of rats in sub-acute oral toxicity test

Satellite group**/** Percentage of body weight change of rats in sub-acute oral toxicity test				
	Sex	Control	DC 1500 mg/kg	*P* value
0 day (g)	M (*n* = 5)	229.20 ± 3.70	235.40 ± 3.85	
	F (*n* = 5)	222.20 ± 5.12	221.00 ± 6.67	
Week 1 (%)	M (*n* = 5)	8.38 ± 0.72	8.09 ± 1.21	0.657
	F (*n* = 5)	4.86 ± 0.59	4.90 ± 1.54	0.960
Week 2 (%)	M (*n* = 5)	15.36 ± 1.57	15.13 ± 0.77	0.782
	F (*n* = 5)	7.57 ± 0.66	7.56 ± 1.67	0.994
Week 3 (%)	M (*n* = 5)	19.90 ± 1.34	19.89 ± 1.62	0.988
	F (*n* = 5)	10.09 ± 1.12	9.80 ± 1.68	0.756
Week 4 (%)	M (*n* = 5)	24.45 ± 1.99	24.30 ± 0.83	0.883
	F (*n* = 5)	12.96 ± 0.96	12.77 ± 1.35	0.807
Week 5 (%)	M (*n* = 5)	28.81 ± 2.02	28.48 ± 1.68	0.788
	F (*n* = 5)	15.22 ± 0.71	14.78 ± 1.81	0.631
Week 6 (%)	M (*n* = 5)	34.03 ± 2.50	33.16 ± 2.69	0.612
	F (*n* = 5)	17.28 ± 0.75	16.59 ± 1.65	0.415

Values expressed as a mea*n* ± standard deviation. Sex (male, M and female, F)

*p-value less than 0.05, (*p* < 0.05) significant value

There was no statistically significant difference in ROW between control and DC treated groups of both tests as *p* > 0.05 (Table 3 A and B). No significant different has been shown in Satellite group in both sexes as *p* > 0.05 (Table 4).

**Table 3:** (A and B) Relative organs weight (g%) of rats in acute and sub-acute oral toxicity tests

A		Acute oral toxicity				
	Sex	Control	DC 300 mg/kg	DC 2000 mg/kg		*P* value
Heart	F (*n* = 3)	0.37 ± 0.02	0.35 ± 0.01	0.35 ± 0.03		0.422
Liver	F (*n* = 3)	2.58 ± 0.14	2.60 ± 0.12	2.50 ± 0.13		0.601
Kidney	F (*n* = 3)	0.70 ± 0.02	0.67 ± 0.03	0.68 ± 0.02		0.484
Spleen	F (*n* = 3)	0.18 ± 0.02	0.18 ± 0.02	0.18 ± 0.01		0.952
Lung	F (*n* = 3)	0.49 ± 0.01	0.48 ± 0.02	0.48 ± 0.02		0.874
B		Sub-acute oral toxicity				
	Sex	Control	DC 500 mg/kg	DC 1000 mg/kg	DC 1500 mg/kg	*P* value
Heart	M (*n* = 5)	0.36 ± 0.02	0.35 ± 0.02	0.34 ± 0.02	0.34 ± 0.03	0.757
	F (*n* = 5)	0.37 ± 0.02	0.37 ± 0.03	0.37 ± 0.02	0.38 ± 0.02	0.938
Liver	M (*n* = 5)	2.92 ± 0.15	2.81 ± 0.10	2.87 ± 0.17	2.92 ± 0.14	0.593
	F (*n* = 5)	2.45 ± 0.09	2.38 ± 0.07	2.35 ± 0.05	2.43 ± 0.07	0.114
Kidney	M (*n* = 5)	0.75 ± 0.02	0.75 ± 0.03	0.76 ± 0.02	0.76 ± 0.03	0.930
	F (*n* = 5)	0.69 ± 0.03	0.70 ± 0.02	0.70 ± 0.05	0.72 ± 0.04	0.639
Spleen	M (*n* = 5)	0.19 ± 0.02	0.19 ± 0.02	0.18 ± 0.03	0.19 ± 0.02	0.937
	F (*n* = 5)	0.18 ± 0.02	0.18 ± 0.02	0.18 ± 0.02	0.19 ± 0.02	0.835
Lung	M (*n* = 5)	0.40 ± 0.02	0.40 ± 0.02	0.39 ± 0.02	0.42 ± 0.01	0.241
	F (*n* = 5)	0.49 ± 0.02	0.48 ± 0.02	0.49 ± 0.01	0.50 ± 0.02	0.536

Values expressed as a mea*n* ± standard deviation. Sex (male, M and female, F)

*p-value less than 0.05, (*p* < 0.05) significant value

**Table 4:** Satellite group/ Relative organs weight (g%) of rats in the sub-acute oral toxicity test

Satellite group/ Relative organs weight (g) of rats in the sub-acute oral toxicity test				
	Sex	Control	DC 1500 mg/kg	*P* value
Heart	M	0.34 ± 0.03	0.34 ± 0.02	0.797
	F	0.38 ± 0.01	0.38 ± 0.01	0.493
Liver	M	2.73 ± 0.09	2.76 ± 0.08	0.508
	F	2.59 ± 0.13	2.64 ± 0.12	0.524
Kidney	M	0.76 ± 0.02	0.75 ± 0.02	0.655
	F	0.72 ± 0.03	0.72 ± 0.03	0.696
Spleen	M	0.19 ± 0.01	0.19 ± 0.01	0.370
	F	0.20 ± 0.02	0.20 ± 0.01	0.832
Lung	M	0.40 ± 0.02	0.38 ± 0.02	0.308
	F	0.50 ± 0.02	0.50 ± 0.01	0.722

Values expressed as a mean ± standard deviation. *n* = 5. Sex (male, M and female, F)

*p-value less than 0.05, (*p* < 0.05) significant value

The food consumption of the DC treated groups in both tests was not significantly different compared to the control group measured throughout the study as *p* > 0.05 (Table 5 A and B) as well as in the satellite groups in both sexes as *p* > 0.05 (Table 6).

**Table 5:** (A and B) Food consumption (g) of rats in acute and sub-acute oral toxicity tests

A		Acute oral toxicity				
	Sex	Control	DC 300 mg/kg	DC 2000 mg/kg		*P* value
Week 1	F (*n* = 3)	64.68 ± 2.80	63.43 ± 2.87	59.14 ± 14.67		0.089
Week 2	F (*n* = 3)	66.16 ± 2.89	67.05 ± 5.14	63.74 ± 2.15		0.236
B		Sub-acute oral toxicity				
	Sex	Control	DC 500 mg/kg	DC 1000 mg/kg	DC 1500 mg/kg	*P* value
Week 1	M (*n* = 5)	81.75 ± 1.21	81.15 ± 2.17	80.99 ± 2.55	79.26 ± 2.42	0.189
	F (*n* = 5)	74.87 ± 2.59	72.99 ± 1.63	72.47 ± 2.28	71.55 ± 2.80	0.089
Week 2	M (*n* = 5)	84.52 ± 1.13	83.93 ± 0.93	83.80 ± 1.77	82.59 ± 1.11	0.061
	F (*n* = 5)	78.69 ± 3.26	77.56 ± 3.21	75.99 ± 3.58	74.66 ± 4.64	0.220
Week 3	M (*n* = 5)	88.05 ± 2.54	87.92 ± 2.07	86.10 ± 1.94	85.19 ± 2.58	0.075
	F (*n* = 5)	86.55 ± 3.64	86.15 ± 3.11	85.17 ± 3.75	83.21 ± 3.68	0.320
Week 4	M (*n* = 5)	91.84 ± 1.60	91.08 ± 0.79	90.30 ± 1.26	90.23 ± 1.11	0.069
	F (*n* = 5)	88.69 ± 3.66	87.35 ± 3.26	87.75 ± 3.32	87.04 ± 2.77	0.798

Values expressed as a mea*n* ± standard deviation. Sex (male, M and female, F)

*p-value less than 0.05, (*p* < 0.05) significant value

**Table 6:** Satellite group/ Food consumption (g) of rats in the sub-acute oral toxicity test

Satellite group/ food consumption in oral sub-acute toxicity test				
	Sex	Control	DC 1500 mg/kg	*P* value
Week 1	M (*n* = 5)	81.92 ± 1.44	79.30 ± 3.81	0.113
	F (*n* = 5)	73.05 ± 3.11	71.26 ± 1.96	0.221
Week 2	M (*n* = 5)	84.60 ± 2.38	82.68 ± 1.56	0.099
	F (*n* = 5)	73.68 ± 2.27	72.77 ± 1.93	0.435
Week 3	M (*n* = 5)	89.75 ± 1.96	87.72 ± 1.69	0.059
	F (*n* = 5)	81.89 ± 3.76	78.62 ± 4.60	0.170
Week 4	M (*n* = 5)	91.96 ± 0.66	91.07 ± 0.93	0.061
	F (*n* = 5)	83.55 ± 2.00	82.43 ± 1.59	0.265
Week 5	M (*n* = 5)	92.96 ± 1.63	91.87 ± 1.80	0.256
	F (*n* = 5)	85.81 ± 1.98	83.92 ± 3.91	0.179
Week 6	M (*n* = 5)	101.90 ± 3.70	100.25 ± 2.85	0.366
	F (*n* = 5)	86.55 ± 3.82	83.07 ± 4.73	0.155

Values expressed as a mea*n* ± standard deviation. Sex (male, M and female, F)

*p-value less than 0.05, (*p* < 0.05) significant value

The water intake of the control and DC treated groups in acute oral toxicity test showed no significant difference as *p* > 0.05 (Table 7 A) while in the sub-acute oral toxicity test a significant difference has been demonstrated between the control and DC treated groups as *p* < 0.05 (Table 7 B). A post hoc Tukey test showed significant differences between the DC treated (male and female) and control groups as shown in Table 8 as *p* < 0.05. Similarly, a significant difference has been shown in Satellite groups between the DC treated group and the control group in both sexes as *p* < 0.05 (Table 9).

**Table 7:** (A and B) Water intake (ml) of rats in the acute and sub-acute oral toxicity tests

A		Acute oral toxicity				
	Sex	Control	DC 300 mg/kg	DC 2000 mg/kg		*P* value
Week 1	F (*n* = 3)	102.56 ± 1.27	104.03 ± 1.78	104.34 ± 2.12		0.157
Week 2	F (*n* = 3)	102.54 ± 0.97	104.00 ± 1.77	103.93 ± 2.01		0.199
B		Sub-acute oral toxicity				
	Sex	Control	DC 500 mg/kg	DC 1000 mg/kg	DC 1500 mg/kg	*P* value
Week 1	M (*n* = 5)	123.18 ± 1.39	128.09 ± 2.34	128.03 ± 1.91	127.40 ± 2.11	0.000*
	F (*n* = 5)	122.39 ± 0.42	125.51 ± 0.50	125.48 ± 0.37	125.46 ± 0.53	0.000*
Week 2	M (*n* = 5)	124.06 ± 1.17	127.31 ± 1.50	127.44 ± 1.48	127.97 ± 1.85	0.000*
	F (*n* = 5)	123.33 ± 0.55	125.68 ± 0.45	125.99 ± 0.41	125.87 ± 0.41	0.000*
Week 3	M (*n* = 5)	125.23 ± 0.96	127.99 ± 1.33	127.98 ± 1.80	127.86 ± 1.69	0.004*
	F (*n* = 5)	124.44 ± 0.49	127.29 ± 0.66	127.12 ± 0.61	127.16 ± 0.77	0.000*
Week 4	M (*n* = 5)	125.89 ± 0.78	128.29 ± 1.95	128.54 ± 1.22	128.34 ± 1.61	0.007*
	F (*n* = 5)	124.99 ± 0.50	127.28 ± 0.86	127.36 ± 0.63	127.56 ± 0.61	0.000*

Values expressed as a mea*n* ± standard deviation. Sex (male, M and female, F)

*p-value less than 0.05, (*p* < 0.05) significant value. Numbers in bold indicate a statistically significant difference

**Table 8:** Tukey test of water intake (ml) of male and female rats in sub-acute oral toxicity test

Dependent variable	(I) water intake	(J) water intake	Mean difference (I-J) in male rat	*P* value	Mean difference (I-J) in female rat	*P* value
Week 1	Control	DC 500 mg**/**kg	−4.91 ± 1.05	0.001*	−3.12 ± 0.24	0.000*
		DC 1000 mg**/**kg	−4.86 ± 1.05	0.001*	−3.09 ± 0.24	0.000*
		DC 1500 mg**/**kg	−4.23 ± 1.05	0.003*	−3.07 ± 0.24	0.000*
Week 2	Control	DC 500 mg**/**kg	−3.25 ± 0.81	0.003*	−2.35 ± 0.25	0.000*
		DC 1000 mg**/**kg	−3.38 ± 0.81	0.002*	−2.67 ± 0.25	0.000*
		DC 1500 mg**/**kg	−3.91 ± 0.81	0.000*	−2.54 ± 0.25	0.000*
Week 3	Control	DC 500 mg**/**kg	−2.77 ± 0.79	0.009*	−2.85 ± 0.34	0.000*
		DC 1000 mg**/**kg	−2.75 ± 0.79	0.010*	−2.68 ± 0.34	0.000*
		DC 1500 mg**/**kg	−2.63 ± 0.79	0.014*	−2.72 ± 0.34	0.000*
Week 4	Control	DC 500 mg**/**kg	−2.40 ± 0.78	0.025*	−2.29 ± 0.35	0.000*
		DC 1000 mg**/**kg	−2.65 ± 0.78	0.012*	−2.37 ± 0.35	0.000*
		DC 1500 mg**/**kg	−2.45 ± 0.78	0.021*	−2.57 ± 0.35	0.000*

Values expressed as a mean ± Standard Error. *n* = 5

*p-value less than 0.05, (*p* < 0.05) significant value. Numbers in bold indicate a statistically significant difference

**Table 9:** Satellite group/ Water intake (ml) of rats in the sub-acute oral toxicity test at each week

Satellite group**/** Water intake (ml) of rats in the sub-acute oral toxicity test at each week				
	Sex	Control	DC 1500 mg/kg	*P* value
Week 1	M	124.39 ± 0.41	125.86 ± 0.85	0.001*
	F	121.24 ± 1.79	123.59 ± 1.96	0.037*
Week 2	M	124.87 ± 0.64	127.14 ± 1.09	0.000*
	F	123.33 ± 1.85	125.03 ± 0.76	0.044*
Week 3	M	126.40 ± 0.87	128.30 ± 1.37	0.009*
	F	123.80 ± 0.95	125.80 ± 1.00	0.002*
Week 4	M	127.48 ± 0.95	128.89 ± 1.21	0.032*
	F	124.53 ± 1.10	125.94 ± 1.01	0.027*
Week 5	M	128.38 ± 1.11	129.03 ± 0.86	0.244
	F	125.68 ± 0.99	125.97 ± 0.68	0.538
Week 6	M	128.94 ± 1.28	129.30 ± 1.34	0.620
	F	126.48 ± 0.90	126.58 ± 0.68	0.825

Values expressed as a mean ± standard deviation. *n* = 5. Sex (male, M and female, F)

*p-value less than 0.05, (*p* < 0.05) significant value. Numbers in bold indicate a statistically significant difference

### Effect of DC extract on hematological parameters in acute and sub-acute oral toxicity tests

A raw data of hematological parameters, is available in the Additional file 1.

The hematological profile of control and DC treated groups summarised in Table 10 (A and B). The results concluded that all hematological parameters such as hemoglobin (HGB) and total white blood cell count are within the normal range in both control and DC treated groups. In ANOVA test, there is no significant association between the groups in both acute and sub-acute toxicity tests as *p >* 0.05. In the satellite groups, there was no significant difference showed in both sexes as *p >* 0.05 (Table 11).

**Table 10:** (A and B) Hematological parameters of the rats in acute and sub-acute oral toxicity tests

A	Acute oral toxicity					
Hematological Parameters	Sex	Control	DC 300 mg/kg	DC2000 mg/kg		*P* value
HGB (g/L)	F (*n* = 3)	153.00 ± 10.00	145.50 ± 9.50	149.33 ± 17.95		0.789
WBC (10^9/L)	F (*n* = 3)	6.83 ± 0.23	7.77 ± 0.38	8.05 ± 0.75		0.057
Neutrophil (10^9/L)	F (*n* = 3)	0.55 ± 0.13	0.56 ± 0.07	0.58 ± 0.14		0.961
Lymphocyte (10^9/L)	F (*n* = 3)	6.39 ± 0.87	6.72 ± 1.15	7.29 ± 0.52		0.498
Monocyte (10^9/L)	F (*n* = 3)	0.14 ± 0.03	0.15 ± 0.02	0.18 ± 0.3		0.228
Eosinophil (10^9/L)	F (*n* = 3)	0.08 ± 0.02	0.10 ± 0.02	0.11 ± 0.02		0.125
Basophil (10^9/L)	F (*n* = 3)	0.02 ± 0.01	0.03 ± 0.02	0.03 ± 0.02		0.531
B	Sub-acute oral toxicity					
Hematological Parameters	Sex	Control	DC 500 mg/kg	DC1000 mg/kg	DC1500 mg/kg	*P* value
HGB (g/L)	M (*n* = 5)	149.40 ± 6.47	148.80 ± 5.40	150.40 ± 12.72	156.80 ± 12.91	0.575
	F (*n* = 5)	156.40 ± 5.81	148.80 ± 7.82	150.60 ± 3.85	153.40 ± 5.81	0.243
WBC (10^9/L)	M (*n* = 5)	9.22 ± 1.03	9.30 ± 2.45	9.46 ± 1.33	9.56 ± 3.67	0.996
	F (*n* = 5)	6.86 ± 0.59	7.40 ± 1.15	7.38 ± 0.93	7.82 ± 0.81	0.431
Neutrophil (10^9/L)	M (*n* = 5)	0.98 ± 0.12	1.01 ± 0.16	1.03 ± 0.18	1.14 ± 0.30	0.626
	F (*n* = 5)	0.81 ± 0.21	0.77 ± 0.11	0.87 ± 0.17	0.89 ± 0.14	0.646
Lymphocyte (10^9/L)	M (*n* = 5)	9.66 ± 2.12	9.64 ± 1.67	10.39 ± 1.99	10.77 ± 2.08	0.753
	F (*n* = 5)	8.22 ± 1.07	8.44 ± 1.22	8.67 ± 1.00	9.20 ± 1.14	0.564
Monocyte (10^9/L)	M (*n* = 5)	0.16 ± 0.02	0.15 ± 0.02	0.17 ± 0.04	0.19 ± 0.04	0.411
	F (*n* = 5)	0.17 ± 0.03	0.16 ± 0.03	0.18 ± 0.02	0.18 ± 0.03	0.623
Eosinophil (10^9/L)	M (*n* = 5)	0.08 ± 0.02	0.09 ± 0.02	0.10 ± 0.02	0.10 ± 0.03	0.388
	F (*n* = 5)	0.08 ± 0.01	0.09 ± 0.02	0.07 ± 0.03	0.10 ± 0.02	0.215
Basophil (10^9/L)	M (*n* = 5)	0.06 ± 0.2	0.04 ± 0.03	0.04 ± 0.03	0.04 ± 0.03	0.537
	F (*n* = 5)	0.02 ± 0.02	0.03 ± 0.02	0.03 ± 0.02	0.04 ± 0.02	0.397

Values expressed as a mea*n* ± standard deviation. Sex (male, M and female, F)

*p-value less than 0.05, (*p* < 0.05) significant value

**Table 11:** Hematological parameters in sub-acute oral toxicity test in Satellite group

Satellite group/ Hematological parameters in sub-acute oral toxicity test				
	Sex	Control	DC 1500 mg/kg	*P* value
HGB (g/L)	M	152.40 ± 6.80	153.20 ± 7.46	0.863
	F	155.00 ± 6.82	154.80 ± 5.97	0.961
WBC (10^9/L)	M	9.30 ± 1.36	10.76 ± 1.23	0.112
	F	6.70 ± 0.72	6.74 ± 0.60	0.926
Neutrophil (10^9/L)	M	1.08 ± 0.13	1.31 ± 0.23	0.084
	F	1.25 ± 0.11	1.33 ± 0.11	0.295
Lymphocyte (10^9/L)	M	9.77 ± 1.07	11.25 ± 1.41	0.098
	F	9.29 ± 0.95	9.31 ± 0.70	0.977
Monocyte (10^9/L)	M	0.21 ± 0.06	0.23 ± 0.07	0.649
	F	0.22 ± 0.05	0.23 ± 0.03	0.773
Eosinophil (10^9/L)	M	0.10 ± 0.01	0.10 ± 0.02	0.856
	F	0.09 ± 0.02	0.10 ± 0.03	0.596
Basophil (10^9/L)	M	0.03 ± 0.02	0.04 ± 0.03	0.636
	F	0.02 ± 0.01	0.03 ± 0.01	0.545

Values expressed as a mean ± standard deviation. *n* = 5. Sex (male, M and female, F). *p-value less than 0.05, (*p* < 0.05) significant value

### Effect of DC extract on serum biochemical parameters in acute and sub-acute oral toxicity tests

A raw data of biochemical parameters, is available in the Additional file 1.

The data on biochemical parameters in control and DC treated groups of the acute oral toxicity test presented in Table 12. There was no significant difference shown in the biochemical parameters between groups as *p* > 0.05.

**Table 12:** Biochemical parameters of the rats in acute oral toxicity test

Biochemical parameters	Sex	Groups			*P* value
		Control	DC 300 mg/kg	DC 2000 mg/kg	
Urea (mmol/L)	F	3.80 ± 0.53	4.00 ± 0.62	4.13 ± 0.29	0.727
Creatinine (umol/L)	F	32.67 ± 1.53	32.00 ± 4.58	31.67 ± 1.53	0.920
Albumin (g/L)	F	40.67 ± 4.04	37.67 ± 3.51	36.67 ± 1.53	0.350
Globulin (g/L)	F	24.00 ± 1.00	22.33 ± 2.08	20.00 ± 2.65	0.128
Total bilirubin (umol/L)	F	2.00 ± 0.00	1.00 ± 0.00	1.00 ± 0.00	–
Conjugate bilirubin (umol/L)	F	1.00 ± 0.00	1.00 ± 0.00	1.00 ± 0.00	–
ALP (U/L)	F	166.33 ± 4.73	164.67 ± 6.03	177.33 ± 7.02	0.081
ALT (U/L)	F	24.67 ± 1.53	25.67 ± 1.15	26.67 ± 1.53	0.296
AST (U/L)	F	96.00 ± 9.17	99.67 ± 7.57	107.33 ± 3.06	0.216

Values expressed as a mean ± standard deviation, *n* = 3

*p-value less than 0.05, (*p* < 0.05) significant value

The data on biochemical parameters in control and DC treated groups of sub-acute oral toxicity presented in Table 13. There was no significant difference shown in the biochemical parameters between the groups in both sexes (male and female rat) as well as in the satellite groups as *p* > 0.05 (Table 14).

**Table 13:** Biochemical parameters of the rats in sub-acute oral toxicity test

Biochemical parameters	Groups					*P* value
	Sex	Control	DC 500 mg/kg	DC 1000 mg/kg	DC 1500 mg/kg	
Urea (mmol/L)	M	3.76 ± 0.59	3.92 ± 0.34	4.14 ± 0.38	4.18 ± 0.51	0.466
	F	3.90 ± 0.74	4.06 ± 0.44	3.97 ± 0.69	4.16 ± 1.24	0.963
Creatinine (umol/L)	M	24.20 ± 4.15	24.00 ± 2.55	23.60 ± 6.91	27.20 ± 4.15	0.615
	F	28.60 ± 3.05	28.40 ± 2.70	27.40 ± 2.70	28.80 ± 1.92	0.839
Albumin (g/L)	M	35.00 ± 2.24	34.60 ± 1.14	36.20 ± 5.26	34.60 ± 1.67	0.817
	F	35.00 ± 1.58	34.60 ± 2.40	36.20 ± 2.17	34.00 ± 2.55	0.470
Globulin (g/L)	M	20.60 ± 1.14	21.00 ± 1.58	21.20 ± 1.48	21.20 ± 1.30	0.890
	F	22.40 ± 1.14	21.80 ± 1.10	22.80 ± 1.30	21.20 ± 1.48	0.245
Total bilirubin (umol/L)	M	1.00 ± 0.00	1.00 ± 0.00	1.00 ± 0.00	1.00 ± 0.00	–
	F	2.00 ± 0.00	2.00 ± 0.00	2.00 ± 0.00	2.00 ± 0.00	–
Conjugate bilirubin (umol/L)	M	1.40 ± 1.14	1.00 ± 0.00	0.40 ± 0.55	1.00 ± 1.22	0.379
	F	1.00 ± 0.00	1.00 ± 0.00	1.00 ± 0.00	1.00 ± 0.00	–
ALP (U/L)	M	216.20 ± 16.99	218.40 ± 12.70	222.40 ± 18.51	236.40 ± 12.74	0.203
	F	204.20 ± 14.64	210.80 ± 29.52	209.60 ± 23.70	197.60 ± 16.33	0.769
ALT (U/L)	M	29.60 ± 3.29	29.40 ± 1.52	29.60 ± 2.30	32.00 ± 2.83	0.356
	F	23.40 ± 3.21	23.60 ± 3.05	25.40 ± 3.36	26.80 ± 1.64	0.243
AST (U/L)	M	104.80 ± 6.69	106.00 ± 3.94	105.40 ± 5.55	109.00 ± 4.95	0.623
	F	99.60 ± 7.40	103 ± 2.30	103.60 ± 3.44	104.60 ± 2.41	0.320

Values expressed as a mean ± standard deviation, *n* = 5. Sex (male, M and female, F)

*p-value less than 0.05, (*p* < 0.05) significant value

**Table 14:** Biochemical parameters of the rats in satellite group for subacute oral toxicity test

Biochemical parameters	Satellite group			*P* value
	Sex	Control	DC 1500 mg/kg	
Urea (mmol/L)	M	3.78 ± 0.34	3.92 ± 0.48	0.608
	F	3.96 ± 0.70	4.06 ± 0.17	0.765
Creatinine (umol/L)	M	25..00 ± 3.87	26.40 ± 3.78	0.579
	F	29.40 ± 3.05	27.20 ± 3.96	0.354
Albumin (g/L)	M	35.20 ± 1.30	34.40 ± 1.67	0.423
	F	34.20 ± 2.77	32.40 ± 3.36	0.382
Globulin (g/L)	M	20.20 ± 0.84	19.40 ± 1.34	0.290
	F	22.00 ± 1.58	21.20 ± 1.30	0.408
Total bilirubin (umol/L)	M	1.00 ± 0.00	1.00 ± 0.00	–
	F	2.00 ± 0.00	2.00 ± 0.00	–
Conjugate bilirubin (umol/L)	M	1.00 ± 0.00	1.00 ± 0.00	–
	F	1.00 ± 0.00	1.00 ± 0.00	–
ALP (U/L)	M	223.60 ± 29.98	226.20 ± 28.35	0.891
	F	184.40 ± 29.11	190.40 ± 29.21	0.753
ALT (U/L)	M	31.00 ± 3.39	30.00 ± 3.81	0.673
	F	25.20 ± 1.79	25.60 ± 2.07	0.752
AST (U/L)	M	107.00 ± 6.04	111.40 ± 5.94	0.279
	F	103.40 ± 3.29	105.00 ± 2.74	0.427

Values expressed as a mean ± standard deviation, *n* = 5. Sex (male, M and female, F)

*p-value less than 0.05, (*p* < 0.05) significant value

### Histopathological observation

A histopathological study carried to confirm biochemical findings and to identify any structural changes. Light microscopic examination of the vital organs including liver, kidney, heart, lung and spleen of the rats in all the DC treated and control groups for acute oral toxicity (Fig. 1) and sub-acute oral toxicity (Fig. 2) did not reveal any gross pathological lesions.

**Fig. 1:** Photomicrograph of vital organs in acute oral toxicity (H & E Stain, ×100). Liver: black arrow – portal vein; white arrow – portal triad. Kidney: black arrow – cortex; white arrow – medulla. Heart: black arrow – myocardium; white arrow – blood vessel. Lung: Black arrow – alveoli; white arrow – bronchiole. Spleen: Black arrow – white pulp, white arrow – red pulp

**Fig. 2:** Photomicrograph of vital organs in sub-acute oral toxicity (H & E Stain, × 100). Liver: black arrow – portal vein; white arrow – portal triad. Kidney: black arrow – cortex; white arrow – medulla. Heart: black arrow – myocardium; white arrow – blood vessel. Lung: Black arrow – alveoli; white arrow – bronchiole. Spleen: Black arrow – white pulp, white arrow – red pulp

The photomicrographs of the liver and kidney of the control and DC treated groups as well as of satellite group, both male and female, showed with normal morphological architecture. Under microscopic examination, the liver of DC treated animals showed with normal cellular architecture and binucleation and was without any distortions similar to the control groups. Furthermore, signs of injury, necrosis, congestion, fatty acid accumulation, or hemorrhagic regions around the central vein or sinusoids of the liver not observed. The hepatocytes arranged in cords and clearly visible. The cross-section of the liver showed no lyses in the blood cells, or infiltration of neutrophil, lymphocyte, or macrophage in the acute oral toxicity group and the sub-acute oral toxicity. For the kidneys, histologically there was no morphological change for all DC treated groups. The appearance of the glomerular architecture showed normal similar to the control groups. The glomeruli, distal, and proximal tubules in the kidney appeared normal in both male and female rats. In addition, there was no interstitial and intraglomerular congestion or tubular atrophies. All the nephron cells showed normal and clearly visible nucleoli with no degeneration, bleeding, or necrosis infiltration in acute oral toxicity group as well as in the sub-acute oral toxicity. In both the control and DC treated female and male rats, the heart shows normal cardiac muscle fibers and lungs show a normal alveolar structure with no treatment-related inflammatory response in acute oral toxicity group as well as in the sub-acute oral toxicity. Similarly, normal structure and histology of the spleen also observed in all the rats of acute and sub-acute oral toxicity tests. There is mild congestion seen in the lung, liver, and kidney of the control and DC treated groups of both sexes which were incidental or spontaneous with no relation to DC resin methanol extraction treatment.

Thus, the histopathological evaluations of the selected organs did not reveal any morphological abnormalities that could be attributed to the oral administration of DC resin methanol extract to the rats.

## Discussion

Herbal medicines have acquired greater importance as a substitute to conventional therapy [49]. As the use of medicinal plants increases, screening plant products to assess and evaluate the toxic characteristics of a natural product extract, fraction, or compound consider an initial step [30].

During the evaluation of the toxic characteristics of medicinal plants, an initial assessment of toxic manifestations is one of the initial screening experiments performed with all compounds. In addition, Data from the acute toxicity study may serve as the basis for classification and labelling of the test material [31]. Thus, the current study was assumed to evaluate and focus on the acute and sub-acute toxicity of DC resin methanol extract in an animal model.

The oral route administration is the most useful and normally used one while doing toxicity study. The absorption may be slow; however, this methodology expenses less and is painless to the animals. As the crude extracts administered orally, the animals need to fast before administering the material because food and other chemicals within the digestive system may have an effect on the reaction(s) of the tested materials. All the procedures were performed based on the appropriate OECD guideline [32].

Test method with a starting dose of 300 mg/kg body weight primarily used in situations where the investigator has no information indicating that the test material is likely to be toxic [23]. In this study, the rats in control and DC treated groups administrated with the vehicle and crude extracts, respectively. From the experiment performed, the starting dose of 300 mg/kg body weight has revealed no mortality in the experimental animals. Thus, the next higher dose of 2000 mg/kg body weight selected as described in the OECD Guidelines 423. The rats monitored daily until the last day of the experiment (day 14th) for any toxic signs and mortality. The clinical symptom is one amongst the most important observations to indicate the toxicity effects on organs within the treated groups [7]. During the 14 days of acute toxicity assessment period, all rats orally administrated with DC resin methanol extract at a single dose of 300 mg/kg and 2000 mg/kg showed no obvious signs of distress, and there were no noticeable symptoms of either toxicity or deaths. All of the rats showed no significant changes in wellness parameters. Physical appearance features such as skin, fur, eyes, mucous membrane, salivation, behavioural pattern, the sleep of the animals in control and DC treated groups (300 mg and 2000 mg) of DC extract were found to be normal. Lethargy, tremors, diarrhoea and coma did not occur in any of the animals. Moreover, the body weight of the rats showed an increase in both control and DC treated groups without significant difference seen (Table 1 A); this indicates that the DC resin methanol extract has no adverse effect on the growth of the animals.

This study estimated that DC resin methanol extract does not cause acute toxicity effects and no rat has died. Based on OECD guidelines 423 (Annex 2), the results of this test allow the substance to be ranked and classified according to the Globally Harmonized System of Classification and Labelling of Chemicals. Thus, the DC resin methanol extract can be classified as category 5 with low acute toxicity hazard, which was the lowest toxicity class [23]. Therefore, it can be concluded that DC resin methanol extract is tolerated up to 2000 mg/kg body weight when administered at a single dose. In a like manner, a study performed by R Ramaswamy, N Prathyusha, R Saranya, H Sumathy, K Mohanavalli, R Priya, J Venkhatesh, C Babu, K Manickavasakam and S Thanikachalam [28] using Nuna Kadugu (a Siddha medicine prepared from leaves and fruits of Morinda Pubescens) revealed that Nuna Kadugu can be classified under category-5 when administered at single dose 2000 mg/kg in accordance with Globally Harmonised System of Classification and Labelling of Chemicals, and this provides a direct relevance for protecting human and animal health.

Acute toxicity information is of limited clinical application because cumulative toxic effects do occur even at very low doses. Consequently, multiple dose studies are typically useful in evaluating the safety profile of phytomedicines. Therefore, sub-acute (Repeated dose 28-day oral toxicity) test has been used. Body weight changes are an indicator of adverse side effects [33], and lose more than 20% of the animal body weight is regarded as critical and has been defined as one of the humane endpoints in several international guidelines [34, 35]. In this study, all rats in the vehicle control and DC treated groups were gaining weight; however, there were no significant changes in body weight gain between the groups in a sub-acute oral test at each week (Table 1 B). Moreover, no significant change detected between the groups in both acute and sub-acute oral toxicity test regarding the ROW (Table 3 A and B). In satellite groups, nothing abnormal detected, and no significant difference was showed in body weight gain and ROW (Tables 2 and 4) respectively.

Sub-acute oral toxicity test was conducted to evaluate the adverse effects of test medicinal plant DC resin methanol extract and was carried out to provide information about the possible health threats that probable to arise from sub-acute exposure over a period of time, the possibilities of cumulative effects, and an estimate of the dose at which there is no observed adverse effect. Evaluation of safety margin between different dose level that produces the therapeutic effect and that which produces the adverse effects is necessary. Evaluation of safety is exactly to provide benefit to risk assessment. Animal experimental model is the only method that can assess this matter [36]. Determination of food consumption is an important to study the safety of a product with therapeutic purpose as proper intake of nutrients is essential to the physiological status of the animal and give a good impression of the appropriate response to the treatment [37].

For food consumption, no significant changes observed in all groups (vehicle and DC extract treated groups) in both acute and subacute oral toxicity tests and this reveals that it did not adversely affect the basic metabolic processes of the experimental animals. On the other hand, water intake showed more in the DC resin methanol extract treated groups than the control, with a significant difference showed in sub-acute oral toxicity test (Table 8) and satellite group (Table 9) for both male and female rats during the administration period. This result could be refereed to that DC resin extract can produce vasodilatation (hypotension) due to relaxation of smooth muscles of blood vessels [9] which in turn stimulate thirst and increase water intake [38].

Hematological and biochemistry data play a major role in determining the toxicity induced by drugs [39]. Blood parameters analysis is appropriate to risk evaluation as the hematological system has a higher prognostic value for toxicity [40]. Blood serves as the main medium of transport for many drugs and xenobiotics in the body and for that reason components of the blood exposed to substantial concentrations of toxic compounds. Damage to and destruction of the blood cells are inimical to normal functioning of the body both in humans and animals [41]. In the present study, the hematological parameters data indicated that DC resin methanol extract did not affect blood cells production as there was no significant difference between the groups in acute and sub-acute oral toxicity tests (Table 10 A and B). In the satellite group, no significant difference showed between the two groups (Table 11). The change in hematological parameters was within the normal range as showed elsewhere [39, 42].

Evaluation of Kidney and Liver function is important in the assessment toxicity of plant extracts as both of them are necessary for the survival of an organism [43]. In animal model toxicity studies, the serum level of creatinine remains the most widely used laboratory test to estimate renal function. It kept within a relatively stable range as daily production and renal excretion are continuous in healthy mammals [44]. In the present study, for kidney function test, two serum renal biochemical parameters, namely urea and creatinine were analyzed as previously mentioned [45]. There were no significant changes observed in urea and creatinine levels between the control and all doses of DC resin methanol extract groups in both acute and sub-acute oral toxicity tests.

The enzymatic activity of the liver such as alanine aminotransferase (ALT), aspartate aminotransferase (AST) and alkaline phosphatase (ALP) was studied to evaluate liver malfunctions. Liver enzymes levels are usually raised in acute hepatoxicity but tend to decrease with prolonged intoxication due to damage to the liver [46]. In the present study, there were no significant differences shown in the biochemical analysis in acute and sub-acute oral toxicity test. The level was within normal expected range for the rat species used in this study. Bilirubin formed from the breakdown of hemoglobin in the liver, spleen, and bone marrow. An increase in tissue or serum bilirubin level occurs through increased breakdown of RBC (hemolysis) or in the case of hepatitis or bile duct obstruction (liver damage) [33]. Reduction in serum albumin level may suggest infection or continuous loss of albumin [47]. Thus, the insignificant change in serum concentration of albumin and globulin in control and DC treated groups at all doses used in this study proposed that DC resin methanol extract not do damage in hepatocellular or secretory functions of the liver which in turn indicated non-adverse effects of the tested material. For biochemical analysis, in the satellite group, there was no significant difference has been noted which concluded that the tested material (DC resin methanol extract) would not produce the delayed onset of toxicity.

The assessment of histopathological alterations in organs considered as a basic test in the safety assessment of tested materials [48]. No abnormality observed on gross or histopathological evaluations of organs examined in this study. Histopathological findings of liver, kidney, heart, lung and spleen were normal in all animals that given different doses of DC resin methanol extract in both acute and sub-acute oral toxicity tests.

However, to determine definitely the oral safety dose and to detect any unanticipated variability of DC resin methanol extract a sub-chronic toxicity and genotoxicity studies might be required. Therefore, sub-chronic toxicity should be proceeded based on the oral doses of DC resin methanol extract in sub-acute oral toxicity test.

## Conclusions

In conclusion, according to Globally Harmonised Classification System, DC resin methanol extract can be classified as Category 5. In addition, we may conclude that DC resin methanol extract is well tolerated up to the dose of 1500 mg/kg body weight administered daily for 28 days. DC resin methanol extract did not cause any lethality or produce any serum chemical alteration or important histopathological signs. The present investigation demonstrates, at least in part, the safety of DC resin methanol extract suggesting its promising potential for pharmaceutical uses.

## Additional file

Additional file 1: The raw data of body weight, organ’s weight, food consumption and water intake, and hematological and biochemical parameters of each rat in the acute and subacute oral toxicity tests. (XLSX 43 kb)

## Abbreviations

ALP: Alkaline phosphatase
ALT: Alanine aminotransferase
ANOVA: One-way analysis of variance
AST: Aspartate aminotransferase
DC: *Dracaena cinnabari*
F: Female
HGB: Hemoglobin
kg: Kilogram
M: Male
mg: Milligram
OECD: Organization for economic cooperation and development
ROW: Relative organ’s weight
SD: Sprague-Dawley
WBC: White blood cell
